The article "Bifurcations of a Fractional-Order Four-Neuron Recurrent Neural Network with Multiple Delays" was published in 2022. Journal: Comput Intell Neurosci.

# Bifurcations of a Fractional-Order Four-Neuron Recurrent Neural Network with Multiple Delays

**DOI:** 10.1155/2022/1779582

**Published:** 2022-09-29

**Authors:** Yu Fei, Rongli Li, Xiaofang Meng, Zhouhong Li

**Affiliations:** ^1^School of Statistics and Mathematics, Yunnan University of Finance and Economics, Kunming, Yunnan 650221, China; ^2^Department of Mathematics, Yuxi Normal University, Yuxi, Yunnan 653100, China

## Abstract

This paper investigates the bifurcation issue of fractional-order four-neuron recurrent neural network with multiple delays. First, the stability and Hopf bifurcation of the system are studied by analyzing the associated characteristic equations. It is shown that the dynamics of delayed fractional-order neural networks not only depend heavily on the communication delay but also significantly affects the applications with different delays. Second, we numerically demonstrate the effect of the order on the Hopf bifurcation. Two numerical examples illustrate the validity of the theoretical results at the end.

## 1. Introduction

Recurrent neural network (RNN) is a type of recursive neural network that takes sequence data as input, recurses in the evolution direction of the sequence, and all nodes (recurrent units) are connected in a chain. Till now, several recurrent neural networks (RNNs) have been widely considered in various fields such as signal processing, optimizations control, image processing, robotics, pattern recognitions, and automatic control, so they have attracted extensive attention of researchers in recent years [1–7]. Since the applications of RNNs depend more heavily on dynamical neural networks, quite a few efforts have been undertaken to study their dynamical properties and a large number of useful results have been investigated, including oscillation, stability, bifurcation, synchronization, and chaos of various RNNs [8–14].

As the matter of fact, for some applications of nonlinear dynamical models, time delay has a significant impact, and in addition to affecting stability, it causes oscillations and other unstable phenomena, such as chaos [15]. Communication delays and the response times of neurons are considered key factors in the performance of neural networks, and this is caused by the finite switching speed of amplifiers and the noninstantaneous signal transmission between neurons [16]. In recently years, many scholars have been interested in studying the dynamics of neural networks with such time delays [17–19]. It must be pointed out that exponential stabilization of memristor-based RNNs with disturbance and mixed time delays by periodically intermittent control has been considered by Wang et al. [20]. Using the appropriate Lyapunov–Krasovski functionals and applying matrix inequality approach methods, Zhou [21] discussed the passivity of a class of recurrent neural networks with impulse and multiproportional delays. Zhou and Zhao [22] investigated the exponential synchronization and polynomial synchronization of recurrent neural networks with and without proportional delays. Robust stability analysis of recurrent neural networks is studied in Refs. [23, 24]. Furthermore, time delays are ubiquitous and unavoidable in the real world. Due to the existence of delays, the system can become unstable, and the dynamic behavior of nonlinear systems becomes more difficult. Moreover, since the solution space of the delay dynamical is infinite, it makes the systems more complex and bifurcation occurs. Hence, it is necessary to consider the properties and dynamics of neural networks via delays, such as time delay [25, 26], multiple delays [27, 28] time-varying delays [29, 30], and so on. In 2013, Zhang and Yang [31] studied a four-neuron recurrent neural network with multiple delays, described as follows:

(1) $$\begin{array}{c} \left\{\begin{array}{c} \dot{x_{1}}\left(t\right)=-x_{1}\left(t\right)+f\left(x_{2}\left(t-\tau_{1}\right)\right)\text{,}\\ \dot{x_{2}}\left(t\right)=-x_{2}\left(t\right)+f\left(x_{3}\left(t-\tau_{1}\right)\right)\text{,}\\ \dot{x_{3}}\left(t\right)=-x_{3}\left(t\right)+f\left(x_{4}\left(t-\tau_{1}\right)\right)\text{,}\\ \dot{x_{4}}\left(t\right)=-x_{4}\left(t\right)+\omega_{1}f\left(x_{1}\left(t-\tau_{2}\right)\right)+\omega_{2}f\left(x_{2}\left(t-\tau_{2}\right)\right)+\omega_{3}f\left(x_{3}\left(t-\tau_{2}\right)\right)\text{,} \end{array}\right. \end{array}$$

**C**5(*α*_1_*β*_1_+*α*_2_*β*_2_)/(*α*_1_^2^+*α*_2_^2^) ≠ 0where *x*_*i*_(*t*)(*i*=1,2,3,4) stand for state of the *i*th neuron at time *t*, *ω*_*k*_ ∈ *R*(*k*=1,2,3) are the network parameters or weight, *f*(·) is the connection function between neurons, and *τ*_*j*_ ≥ 0(*j*=1,2) are the communication time delay. By using the distribution of the solutions of the associated characteristic equation, the Hopf bifurcation and local stability of the four-dimensional RNNs with two delays are studied. For more recurrent neural network research results, see references [5, 10, 12, 20].

In more than three centuries, fractional calculus has developed into a classical mathematical concept. Nonlinear dynamics systems have shown that it has an exceptionally important role in generalizing ordinary differentiation and integration to arbitrary noninteger order. Therefore, if we study the effects of the memory and genetics factors, fractional neural network is sometimes more realistic and more general than integer neural networks. In recent years, the application of fractional order neural networks has developed rapidly, and the complex dynamical behaviors of fractional neural networks has become a very important research hot points, such as stability or multistability, Hopf bifurcation, synchronization, chaos, and so on. For instance, in Ref. [32], the multistability of a fractional-order competitive neural networks with delay is investigated by using the fractional calculus and partitioning of state space. In Lu and Xue [33] study, adaptive synchronization is investigated for fractional delayed stochastic neural networks. Yuan and Huang [34] considered the quantitative analysis of fractional-order neural networks with time delay. Udhayakumar and Rajan [35] discussed Hopf bifurcation of a delayed fractional-order octonion-valued neural networks.

We also know that Hopf bifurcations, which include subcritical and supercritical ones, can be used to efficiently design biochemical oscillators. Furthermore, fractional order neural networks with same delay cannot accurately describe the dynamical properties of real world neural networks compared with the ones with different delays. In recent years, some researchers have considered the dynamical behavior of fractional models with time delay [36–48]. In 2019 [49], we also investigated the existence of Hopf bifurcation for four-neuron fractional neural networks with leakage delays. To the best of our knowledge, so far there are few results on the Hopf bifurcation of four-dimensional fractional-order recurrent neural network with multiple delays are reported, and therefore, the study of Hopf bifurcation of fractional-order dynamical systems with multiple delays remains an open problem.

Based on the above motivations, we are dedicated to presenting a theoretical exploration of stability and Hopf bifurcation for a four-neuron fractional-order recurrent neural network with multiple delays in this work. The main contributions can be highlighted as follows:

- A novel delayed fractional-order recurrent neural network with four-neuron and two different delays is studied
- Double main dynamical properties of the fractional-order recurrent neural network with two delays are investigated: stability and oscillation
- The Hopf bifurcation is discussed in terms of delays and order

In the article, we shall give some some lemmas and definitions of fractional-order calculus in Section 2, and models description in Section 3. In Section 4, the local stability of the trivial steady state of delayed fractional-order RNNs is examined by applying the associated characteristic equation. In addition, the authors will care about the Hopf bifurcation of fractional-order RNNs with multiple delays. In Section 5, two numerical examples are provided to demonstrate the theoretical results. The last section gives some conclusions.

## 2. Preliminaries

This section we will give some Caputo definitions and lemma for fractional calculus as a basis for the theoretical analysis and simulation proofs.

**Definition 1 .**

(see [50]). The fractional integral of order *ϕ* for a function f(x) is defined as follows:

(2) $$\begin{array}{c} I^{\phi }f\left(x\right)=\frac{1}{\Gamma \left(\phi \right)}\int_{x_{0}}^{x}{\left(x-s\right)}^{\phi -1}f\left(s\right)ds\text{,} \end{array}$$

where *ϕ* > 0, and Γ(·) is the Gamma function satisfying Γ(*s*)=∫_0_^*∞*^*x*^*s*−1^*e*^−*x*^d*x*.

**Definition 2 .**

(see [50]). Caputo fractional derivative of order *ϕ* for a function *ψ*(x) ∈ C^k^[x_0_, *∞*), R) is defined by

(3) $$\begin{array}{c} D^{\phi }\psi \left(x\right)=\frac{1}{\Gamma \left(n-\phi \right)}\int_{x_{0}}^{x}\frac{\psi^{\left(k\right)}\left(s\right)}{{\left(x-s\right)}^{\phi -k+1}}ds\text{,} \end{array}$$

where *x* ≥ *x*_0_ and *k* − 1 ≤ *ϕ* < *k*, *k* ∈ *N*^+^.

Moreover, when *ϕ* ∈ (0,1), then

(4) $$\begin{array}{c} D^{\phi }\psi \left(x\right)=\frac{1}{\Gamma \left(1-\phi \right)}\int_{x_{0}}^{x}\frac{\psi^{\prime }\left(s\right)}{{\left(x-s\right)}^{\phi }}ds\text{.} \end{array}$$

**Lemma 1 (see [51]).**

Consider the following fractional order autonomous model.

(5) $$\begin{array}{c} D^{\phi }u=Ju,u\left(0\right)=u_{0}\text{,} \end{array}$$

in which 0 < *ϕ* ≤ 1, u ∈ R^k^, and J ∈ R^k×k^. Then the zero solution of the system (5) is asymptotically stable in the Lyapunov sense if all roots *λ*_*i*_ are the system (5) of character equation satisfy |arg(*λ*_i_)| > *ϕπ*/2(i=1,2,…, k), and then each component of the states decays towards 0 like *t*^−*ϕ*^. In addition, this model is stable if and only if |arg(*λ*_i_)| ≥ *ϕπ*/2 and those critical eigenvalues that satisfy |arg(*λ*_i_)|=*ϕπ*/2 have geometric multiplicity one.

## 3. Mathematics Model Elaboration

This article considers the following four-neuron fractional-order recurrent neural network with two delays:

(6) $$\begin{array}{c} \left\{\begin{array}{c} D^{\phi }x_{1}\left(t\right)=-x_{1}\left(t\right)+f\left(x_{2}\left(t-\tau_{1}\right)\right)\text{,}\\ D^{\phi }x_{2}\left(t\right)=-x_{2}\left(t\right)+f\left(x_{3}\left(t-\tau_{1}\right)\right)\text{,}\\ D^{\phi }x_{3}\left(t\right)=-x_{3}\left(t\right)+f\left(x_{4}\left(t-\tau_{1}\right)\right)\text{,}\\ D^{\phi }x_{4}\left(t\right)=-x_{4}\left(t\right)+\omega_{1}f\left(x_{1}\left(t-\tau_{2}\right)\right)+\omega_{2}f\left(x_{2}\left(t-\tau_{2}\right)\right)+\omega_{3}f\left(x_{3}\left(t-\tau_{2}\right)\right)\text{,} \end{array}\right. \end{array}$$

where *ϕ* ∈ (0,1] are fractional order; *x*_*i*_(*t*)(*i* = 1,2,3,4) stand for state variables; *ω*_*i*_(*i* = 1,2,3) denote the connection weights; the function of connecting neurons is denoted by *f*(*x*(·)); and *τ*_1_ and *τ*_2_ are the communication time delays.

**Remark 1 .**

In fact, if *ϕ*=1, the fractional delayed neural networks (6) changes into the general neural network (1).

Accordingly, the main purpose of this article is to investigate the stability and the application of Hopf bifurcations of the neural networks (6) taking different time delays *τ*_1_ and *τ*_2_ as the bifurcation parameters by the method of stability analysis [52]. In addition, the effects of the order on the creation of the Hopf bifurcation for the proposed fractional order neural network with multiple delays are also numerically discussed.

Throughout of this paper, assume that the following condition holds true:

(**C**1)*f*(·) ∈ C(*R*, *R*), *f*(0)=0, *xf*(*x*) > 0, for *x* ≠ 0.

## 4. Main Results

This section chooses *τ*_1_ or *τ*_2_ as a bifurcation parameter to study the stability analysis and Hopf bifurcation for the fractional order RNNs (6) and to study the bifurcation points accurately.

### 4.1. Bifurcation Depending on *τ*_1_ in Equation (6)

In this subsection, we first study the effects of *τ*_1_ on bifurcations of system (6) by establishing *τ*_2_.

Applying Taylor series formula, the following form of equation (6) at the origin is

(7) $$\begin{array}{c} \left\{\begin{array}{c} D^{\phi }x_{1}\left(t\right)=-x_{1}\left(t\right)+m_{1}x_{2}\left(t-\tau_{1}\right)\text{,}\\ D^{\phi }x_{2}\left(t\right)=-x_{2}\left(t\right)+m_{2}x_{3}\left(t-\tau_{1}\right)\text{,}\\ D^{\phi }x_{3}\left(t\right)=-x_{3}\left(t\right)+m_{3}x_{4}\left(t-\tau_{1}\right)\text{,}\\ D^{\phi }x_{4}\left(t\right)=-x_{4}\left(t\right)+m_{4}x_{1}\left(t-\tau_{2}\right)+m_{5}x_{2}\left(t-\tau_{2}\right)+m_{6}x_{3}\left(t-\tau_{2}\right)\text{.} \end{array}\right. \end{array}$$

By applying Laplace transformation, its characteristic equation is given as

(8) $$\begin{array}{c} de\;t\left(\begin{array}{cccc} s^{\phi }+1 & -m_{1}e^{s\tau_{1}} & 0 & 0\\ 0 & s^{\phi }+1 & -m_{2}e^{-s\tau_{1}} & 0\\ 0 & 0 & s^{\phi }+1 & -m_{3}e^{-s\tau_{1}}\\ -m_{4}e^{-s\tau_{2}} & -m_{5}e^{-s\tau_{2}} & -m_{6}e^{-s\tau_{2}} & s^{\phi }+1 \end{array}\right)=0\text{,} \end{array}$$

where *m*_*k*_=*f*′(0)(*k*=1,2,3), *m*_*k*_=*ω*_*j*_*f*′(0)(*j*=1,2,3, *k*=4,5,6).

From (8), we have

(9) $$\begin{array}{c} K_{1}\left(s\right)+K_{2}\left(s\right)e^{-s\tau_{1}}+K_{3}\left(s\right)e^{-2s\tau_{1}}+K_{4}\left(s\right)e^{-3s\tau_{1}}=0\text{,} \end{array}$$

where

(10) $$\begin{array}{c} K_{1}\left(s\right)=s^{4\phi }+4s^{3\phi }+6s^{2\phi }+4s^{\phi }+1\text{,}\\ K_{2}\left(s\right)=-m_{3}m_{6}\left(s^{2\phi }+2s^{\phi }+1\right)e^{-s\tau_{2}}\text{,}\\ K_{3}\left(s\right)=-m_{2}m_{3}m_{5}\left(s^{\phi }+1\right)e^{-s\tau_{2}}\text{,}\\ K_{4}\left(s\right)=-m_{1}m_{2}m_{3}m_{4}e^{-s\tau_{2}}\text{.} \end{array}$$

Multiplying *e*^*sτ*_1_^ and *e*^2*sτ*_1_^ on both sides of equation (9), respectively, we can obtain

(11) $$\begin{array}{c} \left\{\begin{array}{cc} K_{1}\left(s\right)e^{2s\tau_{1}} & +K_{2}\left(s\right)e^{s\tau_{1}}+K_{3}\left(s\right)+K_{4}\left(s\right)e^{-s\tau_{1}}=0\text{,}\\ K_{1}\left(s\right)e^{s\tau_{1}} & +K_{2}\left(s\right)+K_{3}\left(s\right)e^{-s\tau_{1}}+K_{4}\left(s\right)e^{-2s\tau_{1}}=0\text{.} \end{array}\right. \end{array}$$

Let *K*_1_(*s*)=*A*_1_+*iB*_1_, *K*_2_(*s*)=*A*_2_+*iB*_2_, *K*_3_(*s*)=*A*_3_+*iB*_3_, *K*_4_(*s*)=*A*_4_+*iB*_4_, and from equation (9), we have

(12) $$\begin{array}{c} \left\{\begin{array}{c} \left(A_{1}+iB_{1}\right)e^{2s\tau_{1}}+\left(A_{2}+iB_{2}\right)e^{s\tau_{1}}+\left(A_{3}+iB_{3}\right)+\left(A_{4}+iB_{4}\right)e^{-s\tau_{1}}=0\text{,}\\ \left(A_{1}+iB_{1}\right)e^{s\tau_{1}}+\left(A_{2}+iB_{2}\right)+\left(A_{3}+iB_{3}\right)e^{-s\tau_{1}}+\left(A_{4}+iB_{4}\right)e^{-2s\tau_{1}}=0\text{.} \end{array}\right. \end{array}$$

Take *s*=*iw*=*w*(cos*π*/2+*i* sin*π*/2)(*ω* > 0) be a purely imaginary root of equation (11). Apply inserting *s* into equation (11) and separating the imaginary and real parts yields the following equations:

(13) $$\begin{array}{c} \left\{\begin{array}{c} A_{1}\cos\;\left(2\omega \tau_{1}\right)-B_{1}\sin\;\left(2\omega \tau_{1}\right)+\left(A_{2}+A_{4}\right)\cos\;\left(\omega \tau_{1}\right)+\left(B_{4}-B_{2}\right)\sin\;\left(\omega \tau_{1}\right)=-A_{3}\text{,}\\ B_{1}\cos\;\left(2\omega \tau_{1}\right)+A_{1}\sin\;\left(2\omega \tau_{1}\right)+\left(B_{2}+B_{4}\right)\cos\;\left(\omega \tau_{1}\right)+\left(A_{2}-A_{4}\right)\sin\;\left(\omega \tau_{1}\right)=-B_{3}\text{,}\\ A_{1}\cos\;\left(2\omega \tau_{1}\right)-B_{1}\sin\;\left(2\omega \tau_{1}\right)+\left(A_{2}+A_{4}\right)\cos\;\left(\omega \tau_{1}\right)+\left(B_{4}-B_{2}\right)\sin\;\left(\omega \tau_{1}\right)=-A_{3}\text{,}\\ B_{1}\cos\;\left(2\omega \tau_{1}\right)+A_{1}\sin\;\left(2\omega \tau_{1}\right)+\left(B_{2}+B_{4}\right)\cos\;\left(\omega \tau_{1}\right)+\left(A_{2}-A_{4}\right)\sin\;\left(\omega \tau_{1}\right)=-B_{3}\text{.} \end{array}\right. \end{array}$$

Evidently,

(14) $$\begin{array}{c} \left\{\begin{array}{c} \cos\;\left(\omega \tau_{1}\right)=\frac{F_{12}\left(\omega \right)}{F_{11}\left(\omega \right)}=F_{c1}\left(\omega \right)\text{,}\\ \sin\;\left(\omega \tau_{1}\right)=\frac{F_{22}\left(\omega \right)}{F_{21}\left(\omega \right)}=F_{s1}\left(\omega \right)\text{,} \end{array}\right. \end{array}$$

where *A*_1_, *A*_2_, *A*_3_, *A*_4_, *B*_1_, *B*_2_, *B*_3_, *B*_4_, *F*_11_, *F*_12_, *F*_21,_ and *F*_22_ are given Appendix A. Obviously, from fist to second equation of system (14), it can be implied that

(15) $$\begin{array}{c} F_{c1}^{2}\left(\omega \right)+F_{s1}^{2}\left(\omega \right)=1\text{.} \end{array}$$

From equation (13), one can obtain

(16) $$\begin{array}{c} \tau_{1}^{\left(l\right)}=\frac{1}{w}\left[\arccos\frac{F_{12}\left(w\right)}{F_{11}\left(w\right)}+2l\pi \right],l=0,1,2,\ldots \text{.} \end{array}$$

**Remark 2 .**

This is an inhomogeneous system of linear equations (13), and the independent variables are cos (2*ωτ*_1_), sin (2*ωτ*_1_), cos (*ωτ*_1_), sin (*ωτ*_1_), respectively. According Cramer's rule of linear equation, if the coefficient determinant of the system of linear equations is not equal to 0, we can easily solve solutions of linear equations (13). That is, we can obtain cos (*ωτ*_1_) and sin (*ωτ*_1_) or cos (*ω*2*τ*_1_) and sin (2*ωτ*_1_).

Define the bifurcation point of fractional neural network with multiple delays (6) as

(17) $$\begin{array}{c} \tau_{10}^{*}=\min\left\{\tau_{1}^{\left(l\right)}\right\},l=0,1,2,\ldots \text{.} \end{array}$$

If *τ*_1_ vanishes, then equation (9) becomes

(18) $$\begin{array}{c} H_{1}\left(s\right)+H_{2}\left(s\right)e^{-s\tau_{2}}=0\text{,} \end{array}$$

where

(19) $$\begin{array}{c} H_{1}\left(s\right)=s^{4\phi }+{4s}^{3\phi }+{6s}^{2\phi }+{4s}^{\phi }+1\text{,}\\ H_{2}\left(s\right)={{-m}_{3}m_{6}s}^{2\phi }-{{2m}_{3}m_{6}s}^{\phi }-m_{3}m_{6}-{m_{2}m_{3}m_{5}s}^{\phi }-m_{2}m_{3}m_{5}-m_{1}m_{2}m_{3}m_{4}\text{.} \end{array}$$

If *τ*_2_=0, then the equation (18) becomes

(20) $$\begin{array}{c} 0=s^{4\phi }+4s^{3\phi }+6s^{2\phi }+4s^{\phi }+1-m_{3}m_{6}s^{2\phi }-2m_{3}m_{6}s^{\phi }-m_{3}m_{6}\\ -m_{2}m_{3}m_{5}s^{\phi }-m_{2}m_{3}m_{5}-m_{1}m_{2}m_{3}m_{4}\text{.} \end{array}$$

Suppose that all roots *s* of the equation (18) obey Lemma 1, then we get that both roots *λ*_*i*_ in equation (18) have negative real parts.

The imaginary and real parts of *H*_*j*_(*s*)(*j*=1,2) can be denoted by *H*_*j*_^*I*^ an d *H*_*j*_^*R*^, respectively. Multiplying *e*^2*sτ*_2_^ on both sides of equation (18), we can obtain

(21) $$\begin{array}{c} H_{1}\left(s\right)e^{s\tau_{2}}+H_{2}\left(s\right)=0\text{.} \end{array}$$

Also, let *s*=*iv*=*v*(cos*π*/2+*i* sin*π*/2)(*v* > 0) be a purely imaginary root of equation (11) if and only if

(22) $$\begin{array}{c} \left\{\begin{array}{c} H_{1}^{R}\cos\;\left(v\tau_{2}\right)-H_{1}^{I}\sin\;\left(v\tau_{2}\right)=-H_{2}^{R}\text{,}\\ H_{1}^{I}\cos\;\left(v\tau_{2}\right)+H_{1}^{R}\sin\;\left(v\tau_{2}\right)=-H_{2}^{I}\text{.} \end{array}\right. \end{array}$$

This leads to form

(23) $$\begin{array}{c} \left\{\begin{array}{c} \cos\;\left(v\tau_{2}\right)=-\frac{H_{2}^{R}H_{2}^{R}+H_{1}^{I}H_{2}^{I}}{{H_{1}^{R}}^{2}+{H_{1}^{I}}^{2}}=f_{c1}\left(v\right)\text{,}\\ \sin\;\left(v\tau_{1}\right)=-\frac{-H_{2}^{R}H_{1}^{I}+H_{1}^{R}H_{2}^{I}}{{H_{1}^{R}}^{2}+{H_{1}^{R}}^{2}}=f_{s1}\left(v\right)\text{.} \end{array}\right. \end{array}$$

It is not difficult to see that

(24) $$\begin{array}{c} f_{c1}^{2}\left(w\right)+f_{s1}^{2}\left(w\right)=1\text{.} \end{array}$$

Additionally, we will give the following assumptions which hold true.

(**C**2) The equation (24) has at least a positive real root.

From equation (24), the values of*v* can be obtained according to Mathematics software Mathematica 10.0, and then the Hopf bifurcation point *τ*_20_ of fractional order recurrent neural network (6) with *τ*_1_ = 0 can be derived.To demonstrate our main results, we further present the following hypothesis: (**C**3)Υ_1_Ω_1_ + Υ_2_Ω_2_/Ω_1_^2^ + Ω_2_^2^ ≠ 0, where

(25) $$\begin{array}{c} \Upsilon_{1}=w_{0}\left[\begin{array}{c} A_{2}\sin w_{0}\tau_{10}-B_{2}\cos w_{0}\tau_{10}+2\left(A_{3}\sin\;2w_{0}\tau_{10}-B_{2}\cos\;2w_{0}\tau_{10}\right)\\ \left.+3\left(A_{4}\cos\;3w_{0}\tau_{10}+B_{4}\sin\;3w_{0}\tau_{10}\right.\right], \end{array}\right.\\ \Upsilon_{2}=w_{0}\left[\begin{array}{c} A_{2}\cos w_{0}\tau_{10}+B_{2}\sin w_{0}\tau_{10}+2\left(A_{3}\cos\;2w_{0}\tau_{10}+B_{2}\sin\;2w_{0}\tau_{10}\right)\\ \left.+3\left(A_{4}\cos\;3w_{0}\tau_{10}+B_{4}\sin\;3w_{0}\tau_{10}\right.\right], \end{array}\right.\\ \Omega_{1}=A_{1}^{\prime }+\left[A_{2}^{\prime }-\tau_{1}A_{2}\right]\cos w_{0}\tau_{10}+\left[B_{2}^{\prime }-\tau_{1}B_{2}\right]\sin w_{0}\tau_{10}+\left[A_{3}^{\prime }-2\tau_{1}A_{3}\right]\cos\;2w_{0}\tau_{10}+\left[B_{2}^{\prime }-\tau_{1}B_{3}\right]\sin\;2w_{0}\tau_{10}+\left[A_{4}^{\prime }-3\tau_{1}A_{4}\right]\cos\;3w_{0}\tau_{10}+\left[B_{4}^{\prime }-3\tau_{1}B_{4}\right]\sin\;3w_{0}\tau_{10}\text{,}\\ \Omega_{2}=B_{1}^{\prime }+\left[B_{2}^{\prime }-\tau_{1}B_{2}\right]\cos w_{0}\tau_{10}-\left[A_{2}^{\prime }-\tau_{1}A_{2}\right]\sin w_{0}\tau_{10}+\left[B_{3}^{\prime }-2\tau_{1}B_{3}\right]\cos\;2w_{0}\tau_{10}-\left[A_{2}^{\prime }-\tau_{1}A_{3}\right]\sin\;2w_{0}\tau_{10}+\left[B_{4}^{\prime }-3\tau_{1}B_{4}\right]\cos\;3w_{0}\tau_{10}-\left[A_{4}^{\prime }-3\tau_{1}A_{4}\right]\sin\;3w_{0}\tau_{10}\text{.} \end{array}$$

**Lemma 2 .**

Let s(*τ*_1_)=*ν*(*τ*_10_)+iw(*τ*_1_) be a root of equation (9) near *τ*_1_=*τ*_1__j_ satisfying *ν*(*τ*_1__j_)=0, *w*(*τ*_1__j_)=*w*_0_, then the following transversality condition is satisfied.

(26) $$\begin{array}{c} \text{Re}\left[\frac{ds}{d\tau_{1}}\right]{|}_{\left(w=w_{0},\tau_{1}=\tau_{10}\right)}\neq 0\text{.} \end{array}$$

**Proof**

With implicit function theorem, we can differentiate equation (9) with respect to *τ*_1_, and thus we get

(27) $$\begin{array}{c} 0=K_{1}^{\prime }\left(s\right)\frac{ds}{d\tau_{1}}+K_{2}^{\prime }\left(s\right)e^{-s\tau_{1}}\frac{ds}{d\tau_{1}}+K_{2}\left(s\right)e^{-s\tau_{1}}\left(-\tau_{1}\frac{ds}{d\tau_{1}}-s\right)+K_{3}^{\prime }\left(s\right)e^{-2s\tau_{1}}\frac{ds}{d\tau_{1}}\\ +K_{3}\left(s\right)e^{-2s\tau_{1}}\left(-2\tau_{1}\frac{ds}{d\tau_{1}}-2s\right)+K_{4}^{\prime }\left(s\right)e^{-3s\tau_{1}}\frac{ds}{d\tau_{1}}+K_{4}\left(s\right)e^{-3s\tau -1}\left(-3\tau \frac{ds}{d\tau_{1}}-3s\right)\text{.}\\ \frac{ds}{d\tau_{1}}=\frac{\Upsilon \left(s\right)}{\Omega \left(s\right)}\text{,} \end{array}$$

where

(28) $$\begin{array}{c} \Upsilon \left(s\right)=s\left[K_{2}\left(s\right)e^{-s\tau_{1}}+2K_{3}\left(s\right)e^{2-s\tau_{1}}+3K_{4}\left(s\right)e^{-3s\tau_{1}}\right]\text{,}\\ \Omega \left(s\right)=K_{1}^{\prime }\left(s\right)+\left[K_{2}^{\prime }\left(s\right)-\tau_{1}K_{2}\left(s\right)\right]e^{-2s\tau_{1}}+\left[K_{3}^{\prime }\left(s\right)-2\tau_{1}K_{3}\left(s\right)\right]e^{-2s\tau_{1}}\\ +\left[K_{4}^{\prime }\left(s\right)-3\tau_{1}K_{4}\left(s\right)\right]e^{-3s\tau_{1}}\text{.} \end{array}$$

We further suppose that Υ_1_ and Υ_2_ are the real and imaginary parts of Υ(*s*), respectively, and Ω_1_ and Ω_2_ are the real and imaginary parts of Ω(*s*), respectively, then

(29) $$\begin{array}{c} \text{Re}\left[\frac{ds}{d\tau }\right]{|}_{\left(\tau =\tau_{0}^{*},w=w_{0}^{*}\right)}=\frac{\Upsilon_{1}\Omega_{1}+\Upsilon_{2}\Omega_{2}}{\Omega_{1}^{2}+\Omega_{2}^{2}}\text{.} \end{array}$$

From (**C**3), we conclude that the transversality condition holds true. This completes the proof of Lemma 2.

From the above investigation, we can obtain the following results.

**Theorem 1 .**

assumptions (**C**1)–(**C**3) hold true, then the following results can be given:

- The zero equilibrium point of fractional order four-neuron recurrent neural network with multiple delays (6) is asymptotically stable when *τ*_1_ ∈ [0, *τ*_10_^*∗*^).
- If *τ*_1_ ∈ [0, *τ*_10_^*∗*^), then fractional order four neurons recurrent neural network with multiple delays (6) causes Hopf bifurcation at the origin when *τ*_1_=*τ*_10_^*∗*^. That is, a branch of periodic solutions can bifurcate from the zero equilibrium point at *τ*_1_=*τ*_10_^*∗*^.

### 4.2. Bifurcation Depending on *τ*_2_ in Equation (6)

As in the previous subsection, next we change another delay *τ*_2_ to the bifurcation parameter to account for the bifurcation of the model (6). It is hard to point out that equation (8) changes as follows:

(30) $$\begin{array}{c} q_{1}\left(s\right)+q_{2}\left(s\right)e^{-s\tau_{2}}=0\text{,} \end{array}$$

where

(31) $$\begin{array}{c} q_{1}\left(s\right)=1+4s^{2\phi }+6s^{2\phi }+4s^{3\phi }+s^{4\phi }\text{,}\\ q_{2}\left(s\right)=-m_{3}m_{6}\left(1+2s^{\phi }+s^{2\phi }\right)e^{-s\tau_{1}}-m_{2}m_{3}m_{5}\left(1+s^{\phi }\right)e^{-2s\tau_{1}}-m_{1}m_{2}m_{3}m_{4}e^{-3s\tau_{1}}\text{.} \end{array}$$

Multiplying *e*^2*sτ*_2_^ on both sides of equation (30), we can obtain

(32) $$\begin{array}{c} q_{1}\left(s\right)e^{s\tau_{2}}+q_{2}\left(s\right)=0\text{.} \end{array}$$

Suppose *q*_1_(*s*)=*a*_1_+*ib*_1_ and *q*_2_(*s*)=*a*_2_+*ib*_2_, and from equation (32), we have

(33) $$\begin{array}{c} \left(a_{1}+ib_{1}\right)e^{s\tau_{2}}+a_{2}+ib_{2}=0\text{,} \end{array}$$

where *a*_1_, *a*_2_, *b*_1_, *b*_2_ are given in Appendix B.

Take $s=i\tilde{w}=\tilde{w}\left(\cos\pi /2+i\sin\pi /2\right)\left(\tilde{\omega }>0\right)$ as a root of equation (33) if and only if

(34) $$\begin{array}{c} \left\{\begin{array}{c} a_{1}\cos\;\left(\tilde{w}\tau_{2}\right)-b_{1}\sin\;\left(\tilde{w}\tau_{2}\right)=-a_{2}\text{,}\\ b_{1}\cos\;\left(\tilde{w}\tau_{2}\right)+a_{1}\sin\;\left(\tilde{w}\tau_{2}\right)=-b_{2}\text{,} \end{array}\right. \end{array}$$

that is,

(35) $$\begin{array}{c} \left\{\begin{array}{c} \cos\tilde{w}\tau_{2}=-\frac{a_{1}a_{2}+b_{1}b_{2}}{a_{1}^{2}+b_{1}^{2}}=\rho \left(\tilde{w}\right)\text{,}\\ \sin\tilde{w}\tau_{2}=-\frac{-a_{2}b_{1}+a_{1}b_{2}}{a_{1}^{2}+b_{1}^{2}}=\varrho \left(\tilde{w}\right)\text{.} \end{array}\right. \end{array}$$

It is simple to derive the following equation.

(36) $$\begin{array}{c} \rho^{2}\left(\tilde{w}\right)+\varrho^{2}\left(\tilde{w}\right)=1\text{.} \end{array}$$

From (35), one can obtain

(37) $$\begin{array}{c} \tau_{2}^{\left(l\right)}=\frac{1}{\tilde{w}}\left[\arccos\;\varrho \left(\tilde{w}\right)+2l\pi \right],l=0,1,2,\ldots \text{.} \end{array}$$

The bifurcation point is defined by *ω*_*k*_(*k*=1,2,3)(**C**3)(Υ_1_Ω_1_+Υ_2_Ω_2_)(Ω_1_^2^+Ω_2_^2^) ≠ 0

(38) $$\begin{array}{c} \tau_{20}^{*}=\min\left\{{\tilde{\tau }}_{2}^{\left(l\right)}\right\},l=0,1,2,\ldots \text{.} \end{array}$$

**C**5(*α*_1_*β*_1_+*α*_2_*β*_2_)/(*α*_1_^2^+*α*_2_^2^) ≠ 0 here *τ*_2_^*l*^is defined by equation (38)

If *τ*_2_=0, then the equation (32) becomes

(39) $$\begin{array}{c} M_{1}\left(s\right)+M_{2}\left(s\right)e^{-s\tau_{1}}+M_{3}\left(s\right)e^{-2s\tau_{1}}+M_{4}\left(s\right)e^{-3s\tau_{1}}=0\text{,} \end{array}$$

where

(40) $$\begin{array}{c} M_{1}\left(s\right)=1+4s^{\phi }+6s^{2\phi }+4s^{3\phi }+s^{4\phi }\text{,}\\ M_{2}\left(s\right)=-m_{3}m_{6}\left(1+2s^{\phi }+s^{2\phi }\right)\\ M_{3}\left(s\right)=-m_{2}m_{3}m_{5}\left(1+s^{\phi }\right)\text{,}\\ M_{4}\left(s\right)=-m_{1}m_{2}m_{3}m_{4}\text{.} \end{array}$$

Assume that all roots *s* of equation (39) observe Lemma 1, then we get that both roots of equation (39) have negative real parts.

The imaginary and real parts of *M*_*i*_(*s*)(*i* = 1,2,3,4) can be expressed as *M*_*i*_^*l*^ an d *M*_*i*_^*R*^, respectively. Multiplying both sides of the equation (39) by *e*^2*sτ*_1_^ and *e*^*sτ*_1_^ yields

(41) $$\begin{array}{c} \left\{\begin{array}{c} M_{1}\left(s\right)e^{2s\tau_{1}}+M_{2}\left(s\right)e^{s\tau_{1}}+M_{3}\left(s\right)+M_{4}\left(s\right)e^{-s\tau_{1}}=0\text{,}\\ M_{1}\left(s\right)e^{s\tau_{1}}+M_{2}\left(s\right)+M_{3}\left(s\right)e^{-s\tau_{1}}+M_{4}\left(s\right)e^{-2s\tau_{1}}=0\text{.} \end{array}\right. \end{array}$$

Let $s=i\tilde{v}=\tilde{v}\left(\cos\pi /2+i\;\sin\pi /2\right)\left(\tilde{v}>0\right)$ be a solution of equation (41). Substituting *s* into equation (41) and separating the imaginary and real units yields the following equations:

(42) $$\begin{array}{c} \left\{\begin{array}{c} M_{1}^{R}\cos\;\left(2\tilde{v}\tau_{1}\right)-M_{1}^{I}\sin\;\left(2\tilde{v}\tau_{1}\right)+\left(M_{2}^{R}+M_{4}^{R}\right)\cos\;\left(\tilde{v}\tau_{1}\right)+\left(M_{4}^{I}-P_{2}^{I}\right)\sin\;\left(\tilde{v}\tau_{1}\right)=-M_{3}^{R}\text{,}\\ M_{1}^{I}\cos\;\left(2\tilde{v}\tau_{1}\right)+M_{1}^{R}\sin\;\left(2\tilde{v}\tau_{1}\right)+\left(M_{2}^{I}+M_{4}^{I}\right)\cos\;\left(\tilde{v}\tau_{1}\right)+\left(M_{2}^{R}-P_{4}^{R}\right)\sin\;\left(\tilde{v}\tau_{1}\right)=-M_{3}^{I}\text{,}\\ P_{1}^{R}\cos\;\left(2\tilde{v}\tau_{1}\right)-M_{1}^{I}\sin\;\left(2\tilde{v}\tau_{1}\right)+\left(M_{2}^{R}+P_{4}^{R}\right)\cos\;\left(\tilde{v}\tau_{1}\right)+\left(M_{4}^{I}-P_{2}^{I}\right)\sin\;\left(\tilde{v}\tau_{1}\right)=-M_{3}^{R}\text{,}\\ P_{1}^{I}\cos\;\left(2\tilde{v}\tau_{1}\right)+M_{1}^{R}\sin\;\left(2\tilde{v}\tau_{1}\right)+\left(M_{2}^{I}+P_{4}^{R}\right)\cos\;\left(\tilde{v}\tau_{1}\right)+\left(M_{2}^{R}-P_{4}^{R}\right)\sin\;\left(\tilde{v}\tau_{1}\right)=-M_{3}^{I}\text{,} \end{array}\right. \end{array}$$

which lead to

(43) $$\begin{array}{c} \left\{\begin{array}{c} \cos\tilde{v}\tau_{1}=\frac{E_{12}\left(\tilde{v}\right)}{E_{11}\left(\tilde{v}\right)}=C{\left(\tilde{v}\right)}^{2}\text{,}\\ \sin\tilde{v}\tau_{1}=\frac{E_{22}\left(\tilde{v}\right)}{E_{21}\left(\tilde{v}\right)}=S{\left(\tilde{v}\right)}^{2}\text{.} \end{array}\right. \end{array}$$

Obviously, from first and second equation of system (43), we get

(44) $$\begin{array}{c} C{\left(\tilde{v}\right)}^{2}+S{\left(\tilde{v}\right)}^{2}=1\text{.} \end{array}$$

To theoretically gain the sufficient conditions for the Hopf bifurcation, we assume that the following assumptions hold true:

(**C**4) Equation (36) has at least a positive real root.

By means of equation (36), the values of $\tilde{\omega }$ can be obtained according to mathematical software Mathematica 10.0, and then the bifurcation point *τ*_10_ of recullrent fractional four-neuron neural networks (6) with *τ*_2_ = 0 can be derived.As a summary of our main results, we provide the following assumption: (**C**5)*α*_1_*β*_1_ + *α*_2_*β*_2_/*α*_1_^2^ + *α*_2_^2^ ≠ 0, where

(45) $$\begin{array}{c} \alpha_{1}=a_{1}^{\prime }+\left(a_{2}^{\prime }-\tau_{20}a_{2}\right)\cos{\tilde{w}}_{0}\tau_{20}+\left(b_{2}^{\prime }-\tau_{2}b_{2}\right)\sin{\tilde{w}}_{0}\tau_{20}\text{,}\\ \alpha_{2}=b_{1}^{\prime }+\left(b_{2}^{\prime }-\tau_{20}b_{2}\right)\cos{\tilde{w}}_{0}\tau_{20}-\left(a_{2}^{\prime }-\tau_{2}a_{2}\right)\sin{\tilde{w}}_{0}\tau_{20}\text{,}\\ \beta_{1}={\tilde{w}}_{0}\left(a_{2}\sin{\tilde{w}}_{0}\tau_{20}-b_{2}\cos{\tilde{w}}_{0}\tau_{20}\right)\text{,}\\ \beta_{2}={\tilde{w}}_{0}\left(a_{2}\cos{\tilde{w}}_{0}\tau_{20}+b_{2}\sin{\tilde{w}}_{0}\tau_{20}\right)\text{.} \end{array}$$

**Lemma 3 .**

Let $s\left(\tau_{2}\right)=\eta \left(\tau_{2}\right)+i\tilde{w}\left(\tau_{2}\right)$ be a root of equation (9) near *τ*_2_=*τ*_2__j_ satisfying *η*(*τ*_2__j_)=0, $w\left({\tau_{2}}_{j}\right)={\tilde{w}}_{0}$, then we get the following transversality condition

(46) $$\begin{array}{c} \text{Re}\left[\frac{ds}{d\tau_{2}}\right]{|}_{\left(\tilde{w}={\tilde{w}}_{0},\tau_{2}=\tau_{20}\right)}\neq 0\text{.} \end{array}$$

**Proof**

Similar to Lemma 2, by utilizing the implicit function theorem and differentiating (9) with respect to *τ*_2_, we get

(47) $$\begin{array}{c} 0=q_{1}^{\prime }\left(s\right)\frac{ds}{d\tau_{2}}+q_{2}^{\prime }\left(s\right)e^{-s\tau_{2}}\frac{ds}{d\tau_{2}}+q_{2}\left(s\right)e^{-s\tau_{2}}\left(-\tau_{2}\frac{ds}{d\tau_{2}}-s\right),\frac{ds}{d\tau_{2}}=\frac{\beta \left(s\right)}{\alpha \left(s\right)}\text{,} \end{array}$$

where

(48) $$\begin{array}{c} \beta \left(s\right)=sq_{2}\left(s\right)e^{-s\tau_{2}}\text{,}\\ \alpha \left(s\right)=q_{1}^{\prime }\left(s\right)+q_{2}^{\prime }\left(s\right)e^{-s\tau_{2}}-\tau_{2}q_{2}\left(s\right)e^{-s\tau_{2}}\text{.} \end{array}$$

We further suppose that *α*_1_ and *α*_2_ are the real and imaginary units of *α*(*s*), respectively, and *β*_1_ and *β*_2_ are the real and imaginary parts of *β*(*s*), respectively, then we get

(49) $$\begin{array}{c} \text{Re}\left[\frac{ds}{d\tau_{2}}\right]{|}_{\left(\tilde{w}={\tilde{w}}_{0},\tau_{2}=\tau_{20}\right)}=\frac{\alpha_{1}\beta_{1}+\alpha_{2}\beta_{2}}{\alpha_{1}^{2}+\alpha_{2}^{2}}\text{.} \end{array}$$

As a direct consequence of (**C**5), we can conclude that the transversality condition is satisfied. Then the proof of Lemma 3 is complete.

Based on the above analysis, the following conclusions can be drawn.

**Theorem 2 .**

By assuming that assumptions (**C**1), (**C**4), and (**C**5) are valid, the following conditions can be inferred:

- The zero equilibrium point of fractional order four-neuron recurrent neural network with multiple delays (6) is asymptotically stable when *τ*_2_ ∈ [0, *τ*_20_^*∗*^))
- The fractional order four-neuron recurrent neural network with multiple delays (6) experiences a Hopf bifurcation at its origin when *τ*_2_=*τ*_20_^*∗*^; that is, a family of periodic solutions can bifurcate from the zero equilibrium point near *τ*_2_=*τ*_20_^*∗*^

## 5. Numerical Examples

To demonstrate the validity and feasibility of the conclusions reached in this paper, we provide two examples. The simulations were based on a prediction and correction scheme [53] of Adama–Bashforth–Moulton and step-size *h*=0.01.

### 5.1. Example 1

Consider the four-neuron fractional recurrent neural networks with multiple delays as

(50) $$\begin{array}{c} \left\{\begin{array}{c} D^{\phi }x_{1}\left(t\right)=-x_{1}\left(t\right)+f\left(x_{2}\left(t-\tau_{1}\right)\right)\text{,}\\ D^{\phi }x_{2}\left(t\right)=-x_{2}\left(t\right)+f\left(x_{3}\left(t-\tau_{1}\right)\right)\text{,}\\ D^{\phi }x_{3}\left(t\right)=-x_{3}\left(t\right)+f\left(x_{4}\left(t-\tau_{1}\right)\right)\text{,}\\ D^{\phi }x_{4}\left(t\right)=-x_{4}\left(t\right)+\omega_{1}f\left(x_{1}\left(t-\tau_{2}\right)\right)+\omega_{2}f\left(x_{2}\left(t-\tau_{2}\right)\right)+\omega_{3}f\left(x_{3}\left(t-\tau_{2}\right)\right)\text{.} \end{array}\right. \end{array}$$

Choose parameters *ϕ*=0.9, *ω*_1_=2, *ω*_2_=*ω*_3_=−2, action function *f*(·)=tanh(·); therefore, *f*(0)=tanh(0)=0, *f*′(0)=1.

Let the initial values be selected as (*x*_1_(0), *x*_2_(0), *x*_3_(0), *x*_4_(0))=(0.15, −0.14,0.1,0.2) for the system (50). First, taking fixed *τ*_2_ such that *τ*_2_=0.6 by complex computing, we get *ω*_10_=5.23599, and then *τ*_10_=0.312709. Obviously, it is easy to verify that the conditions in Theorem 1 are satisfied. The numerical simulations in Figures 1 and 2 that the zero equilibrium point of system (50) is locally asymptotically stable when *τ*_1_=0.25 < *τ*_10_=0.312709. Moreover, Figures 3 and 4 simulates that the zero equilibrium point of system (50) is unstable, and Hopf bifurcation occurs when *τ*_1_=0.35 > *τ*_10_=0.312709. The bifurcation diagrams are plotted in Figure 5, which illustrates the theoretical results.

### 5.2. Example 2

The same as example 1, let *ϕ*=0.95, and now we consider the following four-neurons fractional current network with double different delays:

(51) $$\begin{array}{c} \left\{\begin{array}{c} D^{0.95}x_{1}\left(t\right)=-x_{1}\left(t\right)+f\left(x_{2}\left(t-\tau_{1}\right)\right)\text{,}\\ D^{0.95}x_{2}\left(t\right)=-x_{2}\left(t\right)+f\left(x_{3}\left(t-\tau_{1}\right)\right)\text{,}\\ D^{0.95}x_{3}\left(t\right)=-x_{3}\left(t\right)+f\left(x_{4}\left(t-\tau_{1}\right)\right)\text{,}\\ D^{0.95}x_{4}\left(t\right)=-x_{4}\left(t\right)+\omega_{1}f\left(x_{1}\left(t-\tau_{2}\right)\right)+\omega_{2}f\left(x_{2}\left(t-\tau_{2}\right)\right)+\omega_{3}f\left(x_{3}\left(t-\tau_{2}\right)\right)\text{.} \end{array}\right. \end{array}$$

Taking *ω*_1_ = 1, *ω*_2_ = *ω*_3_ = −1.5, *ϕ* = 0.95, action function *f*(·) = tanh(·), then *f*(0) = tanh(0) = 0, *f*′(0) = 1, and we first also set *τ*_1_ = 0.8, in the next step, we apply a complex calculation, and it obtains a ${\tilde{\omega }}_{20}=1.02089$ and *τ*_20_ = 0.329454. Thus, Theorem 2 yields that the zero solution (0,0,0,0) of the system (51) is locally asymptotically stable when *τ*_2_ = 0.22 < *τ*_20_, which is simulated in Figures 6 and 7 which describes the impact of fractional order on *τ*_20_. In addition, the zero equilibrium point of the system (51) is unstable, and Hopf bifurcation occurs when *τ*_2_ = 0.38 > *τ*_20_, as shown in Figures 8 and 9. Moreover, the bifurcation diagrams are plotted in Figure 10, which illustrates the theoretical results.

**Remark 3 .**

In fact, in order to better reflect the influence of different time delays at the bifurcation point of the systems (50) and (51), the corresponding bifurcation point *τ*_10_ and *τ*_20_ and *τ*_10_^*∗*^ and *τ*_20_^*∗*^ can be determined by changing the order of *ϕ*. This means that systems (50) and (51) involving different two delays are prone to earlier Hopf bifurcation for some fixed fractional order *ϕ*.

## 6. Conclusion

This paper examines the Hopf bifurcation problem of fractional recurrent neural networks with four neurons and two delays. Using time delay as the bifurcation parameter, several criteria are destabilized in order to ensure the Hopf bifurcation for the fractional four-neuron of recurrent neural networks. Based on our analysis, different communication time delays and order effects have quantitatively changed the dynamic behavior of the system (6). These results can contribute to our understanding of delayed fractional recurrent neural networks as a continuation of the previous work. The results of the simulations are illustrated by two numerical examples.

## Figures and Tables

**Figure 1:** Time responses of system (50) with *ϕ*=0.9, *τ*_1_=0.25 < *τ*_10_=0.312709.

**Figure 2:** Phase diagrams of system (50) with *ϕ*=0.9, *τ*_1_=0.25 < *τ*_10_=0.312709.

**Figure 3:** Time responses of system (50) with *ϕ*=0.9, *τ*_1_=0.36 > *τ*_10_=0.312709.

**Figure 4:** Phase diagrams of system (50) with *ϕ*=0.9, *τ*_1_=0.36 > *τ*_10_=0.312709.

**Figure 5:** Bifurcation diagram of system (50) with *ϕ*=0.9, *τ*_1_=0.36 > *τ*_10_=0.312709.

**Figure 6:** Time responses of system (51) with *ϕ*=0.95, *τ*_1_=0.22 < *τ*_20_=0.329454.

**Figure 7:** Phase diagrams of system (51) with *ϕ*=0.95, *τ*_1_=0.22 < *τ*_20_=0.329454.

**Figure 8:** Time responses of system (51) with *ϕ*=0.95, *τ*_1_=0.38 > *τ*_20_=0.329454.

**Figure 9:** Phase diagrams of system (51) with *ϕ*=0.95, *τ*_1_=0.38 > *τ*_20_=0.329454.

**Figure 10:** Bifurcation diagrams of system (51) with *ϕ*=0.95, *τ*_1_=0.38 > *τ*_20_=0.329454.

## Data Availability

Data sharing not is applicable in this article as no datasets were generated or analysed during the current paper.

## Appendix

### A

(A.1)
$$\begin{array}{c} A_{1}=6\omega^{2\phi }\;\cos\;\left(\pi \phi \right)+4\omega^{3\phi }\;\cos\left(\frac{3\pi \phi }{2}\right)+\omega^{4\phi }\;\cos\;\left(2\pi \phi \right)+4\omega^{\phi }\;\cos\left(\frac{\pi \phi }{2}\right)+1\text{,}\\ B_{1}=6\omega^{2\phi }\;\sin\;\left(\pi \phi \right)+4\omega^{3\phi }\;\sin\left(\frac{3\pi \phi }{2}\right)+\omega^{4\phi }\;\sin\;\left(2\pi \phi \right)+4\omega^{\phi }\;\sin\left(\frac{\pi \phi }{2}\right)\text{,}\\ A_{2}=-m_{3}m_{6}\omega^{2\phi }\;\sin\;\left(\pi \phi \right)\sin\;\left(\omega \tau_{2}\right)-m_{3}m_{6}\omega^{2\phi }\;\cos\;\left(\pi \phi \right)\cos\;\left(\omega \tau_{2}\right)\\ -2m_{3}m_{6}\omega^{\phi }\;\sin\left(\frac{\pi \phi }{2}\right)\sin\;\left(\omega \tau_{2}\right)-2m_{3}m_{6}\omega^{\phi }\;\cos\left(\frac{\pi \phi }{2}\right)\cos\;\left(\omega \tau_{2}\right)-m_{3}m_{6}\cos\;\left(\omega \tau_{2}\right)\text{,}\\ B_{2}=-m_{3}m_{6}\omega^{2\phi }\;\sin\;\left(\pi \phi \right)\cos\;\left(\omega \tau_{2}\right)+m_{3}m_{6}\omega^{2\phi }\;\cos\;\left(\pi \phi \right)\sin\;\left(\omega \tau_{2}\right)\\ -2m_{3}m_{6}\omega^{\phi }\;\sin\left(\frac{\pi \phi }{2}\right)\cos\;\left(\omega \tau_{2}\right)+2m_{3}m_{6}\omega^{\phi }\;\cos\left(\frac{\pi \phi }{2}\right)\sin\;\left(\omega \tau_{2}\right)+m_{3}m_{6}\sin\;\left(\omega \tau_{2}\right)\text{,}\\ A_{3}=-m_{2}m_{3}m_{5}\omega^{\phi }\;\sin\left(\frac{\pi \phi }{2}\right)\sin\;\left(\omega \tau_{2}\right)-m_{2}m_{3}m_{5}\omega^{\phi }\;\cos\left(\frac{\pi \phi }{2}\right)\cos\;\left(\omega \tau_{2}\right)-m_{2}m_{3}m_{5}\cos\;\left(\omega \tau_{2}\right)\text{,}\\ B_{3}=-m_{2}m_{3}m_{5}\omega^{\phi }\;\sin\left(\frac{\pi \phi }{2}\right)\cos\;\left(\omega \tau_{2}\right)+m_{2}m_{3}m_{5}\omega^{\phi }\;\cos\left(\frac{\pi \phi }{2}\right)\sin\;\left(\omega \tau_{2}\right)+m_{2}m_{3}m_{5}\sin\;\left(\omega \tau_{2}\right)\text{,}\\ A_{4}=-m_{1}m_{2}m_{3}m_{4}\cos\;\left(\omega \tau_{2}\right)\text{,}\\ B_{4}=m_{1}m_{2}m_{3}m_{4}\sin\;\left(\omega \tau_{2}\right)\text{,}\\ F_{11}=-B_{4}^{2}\left(A_{1}B_{4}+A_{4}B_{1}\right)\left(A_{1}^{4}-A_{1}^{2}\left(A_{3}^{2}+2A_{4}^{2}-2B_{1}^{2}+B_{3}^{2}+2B_{4}^{2}\right)+2A_{1}\right.\left(A_{2}A_{3}A_{4}\right.\\ +A_{2}B_{3}B_{4}+A_{3}B_{2}B_{4}-A_{4}B_{2}\left.B_{3}\right)-A_{2}^{2}\left(A_{4}^{2}+B_{4}^{2}\right)+2A_{2}B_{1}\left(A_{4}B_{3}-A_{3}B_{4}\right)\\ -A_{3}^{2}B_{1}^{2}+2A_{3}A_{4}B_{1}B_{2}+A_{4}^{4}-2A_{4}^{2}B_{1}^{2}-A_{4}^{2}B_{2}^{2}+2A_{4}^{2}B_{4}^{2}+B_{1}^{4}-B_{1}^{2}B_{3}^{2}\\ -2B_{1}^{2}B_{4}^{2}+2B_{1}B_{2}B_{3}B_{4}-B_{2}^{2}B_{4}^{2}+\left.B_{4}^{4}\right)\text{,}\\ F_{12}=B_{4}\left(-\left(\left(A_{4}^{2}+B_{4}^{2}\right)\right.\left(A_{2}B_{1}+A_{3}B_{4}\right)-\left(A_{1}B_{4}+A_{4}B_{1}\right)\left(A_{2}A_{4}+B_{2}B_{4}\right)\right)\left(A_{1}^{2}\left(B_{1}-B_{3}\right)\right.\\ +\left.A_{1}\left(A_{2}B_{4}-A_{4}B_{2}\right)+B_{1}\left(A_{2}A_{4}-A_{4}^{2}+B_{1}^{2}-B_{1}B_{3}+B_{2}B_{4}-B_{4}^{2}\right)\right)-B_{4}\left(-A_{1}^{2}A_{2}\right.\\ \left.+A_{1}\left(A_{3}A_{4}+B_{3}B_{4}\right)-B_{1}\left(A_{2}B_{1}+A_{3}B_{4}-A_{4}B_{3}\right)\right)\left(B_{4}\left(A_{1}^{2}+B_{1}^{2}-B_{1}B_{3}\right.\right.\\ \left.\left.\left.+B_{4}\left(B_{2}-B_{4}\right)\right)-A_{3}\left(A_{1}B_{4}+A_{4}B_{1}\right)+A_{1}A_{4}B_{3}+A_{4}^{2}\left(B_{2}-B_{4}\right)\right)\right)\text{,}\\ F_{21}=A_{1}^{4}-A_{1}^{2}\left(A_{3}^{2}+2A_{4}^{2}-2B_{1}^{2}+B_{3}^{2}+2B_{4}^{2}\right)+2A_{1}\left(A_{2}A_{3}A_{4}+A_{2}B_{3}B_{4}+A_{3}B_{2}B_{4}\right.\\ -A_{4}B_{2}\left.B_{3}\right)-A_{2}^{2}\left(A_{4}^{2}+B_{4}^{2}\right)+2A_{2}B_{1}\left(A_{4}B_{3}-A_{3}B_{4}\right)-A_{3}^{2}B_{1}^{2}+2A_{3}A_{4}B_{1}B_{2}\\ +A_{4}^{4}-2A_{4}^{2}B_{1}^{2}-A_{4}^{2}B_{2}^{2}+2A_{4}^{2}B_{4}^{2}+B_{1}^{4}-B_{1}^{2}B_{3}^{2}-2B_{1}^{2}B_{4}^{2}+2B_{1}B_{2}B_{3}B_{4}-B_{2}^{2}B_{4}^{2}+B_{4}^{4}\text{,}\\ F_{22}=A_{1}^{3}\left(-B_{2}\right)+A_{1}^{2}\left(A_{2}\left(B_{1}+B_{3}\right)+A_{3}\left(B_{4}-B_{2}\right)-A_{4}B_{3}\right)+A_{1}\left(A_{2}^{2}\left(-B_{4}\right)+2A_{2}A_{4}B_{2}\right.\\ +A_{3}^{2}B_{4}-2A_{3}A_{4}B_{3}+A_{4}^{2}B_{2}-B_{1}^{2}B_{2}+B_{2}^{2}B_{4}+B_{2}B_{4}^{2}-B_{3}^{2}\left.B_{4}\right)-A_{2}^{2}A_{4}B_{1}\\ +A_{2}\left(A_{4}^{2}\left(B_{3}-B_{1}\right)+B_{1}^{3}+B_{1}^{2}B_{3}-B_{1}B_{4}\left(2B_{2}+B_{4}\right)+B_{3}B_{4}^{2}\right)+A_{3}^{2}A_{4}B_{1}\\ -A_{3}A_{4}^{2}B_{2}-A_{3}A_{4}^{2}B_{4}-A_{3}B_{1}^{2}B_{2}+A_{3}B_{1}^{2}B_{4}+2A_{3}B_{1}B_{3}B_{4}-A_{3}B_{2}B_{4}^{2}-A_{3}B_{4}^{3}\\ +A_{4}^{3}B_{3}-A_{4}B_{1}^{2}B_{3}+A_{4}B_{1}B_{2}^{2}-A_{4}B_{1}B_{3}^{2}+A_{4}B_{3}B_{4}^{2}\text{.} \end{array}$$

### B

(B.1)
$$\begin{array}{c} a_{1}=6{\tilde{\omega }}^{2\phi }\;\cos\;\left(\pi \phi \right)+4{\tilde{\omega }}^{3\phi }\;\cos\left(\frac{3\pi \phi }{2}\right)+{\tilde{\omega }}^{4\phi }\;\cos\;\left(2\pi \phi \right)+4{\tilde{\omega }}^{\phi }\;\cos\left(\frac{\pi \phi }{2}\right)+1\text{,}\\ b_{1}=6{\tilde{\omega }}^{2\phi }\;\sin\;\left(\pi \phi \right)+4{\tilde{\omega }}^{3\phi }\;\sin\left(\frac{3\pi \phi }{2}\right)+{\tilde{\omega }}^{4\phi }\;\sin\;\left(2\pi \phi \right)+4{\tilde{\omega }}^{\phi }\;\sin\left(\frac{\pi \phi }{2}\right)\text{,}\\ a_{2}=-m_{2}m_{3}\left(m_{1}m_{4}\cos\;\left(3\tilde{\omega }\tau_{1}\right)+m_{5}{\tilde{\omega }}^{\phi }\;\sin\left(\frac{\pi \phi }{2}\right)\sin\;\left(2\tilde{\omega }\tau_{1}\right)\right)\\ -m_{2}m_{3}m_{5}\left({\tilde{\omega }}^{\phi }\;\cos\left(\frac{\pi \phi }{2}\right)\cos\;\left(2\tilde{\omega }\tau_{1}\right)+\cos\;\left(2\tilde{\omega }\tau_{1}\right)\right)\\ -m_{3}m_{6}\left({\tilde{\omega }}^{2\phi }\;\sin\;\left(\pi \phi \right)\sin\;\left(\tilde{\omega }\tau_{1}\right)+{\tilde{\omega }}^{2\phi }\;\cos\;\left(\pi \phi \right)\cos\;\left(\tilde{\omega }\tau_{1}\right)\right.\\ \left.+2{\tilde{\omega }}^{\phi }\;\sin\left(\frac{\pi \phi }{2}\right)\sin\;\left(\tilde{\omega }\tau_{1}\right)+2{\tilde{\omega }}^{\phi }\;\cos\left(\frac{\pi \phi }{2}\right)\cos\;\left(\tilde{\omega }\tau_{1}\right)+\cos\;\left(\tilde{\omega }\tau_{1}\right)\right)\text{,}\\ b_{2}=m_{2}m_{3}\left(m_{1}m_{4}\sin\;\left(3\tilde{\omega }\tau_{1}\right)+m_{5}{\tilde{\omega }}^{\phi }\;\sin\left(\frac{\pi \phi }{2}\right)\cos\;\left(2\tilde{\omega }\tau_{1}\right)\right)+m_{2}m_{3}m_{5}\left({\tilde{\omega }}^{\phi }\;\cos\left(\frac{\pi \phi }{2}\right)\right.\\ \times \left.\sin\;\left(2\tilde{\omega }\tau_{1}\right)+\sin\;\left(2\tilde{\omega }\tau_{1}\right)\right)-m_{3}m_{6}\left({\tilde{\omega }}^{2\phi }\;\sin\;\left(\pi \phi \right)\cos\;\left(\tilde{\omega }\tau_{1}\right)-{\tilde{\omega }}^{2\phi }\;\cos\;\left(\pi \phi \right)\sin\;\left(\tilde{\omega }\tau_{1}\right)\right.\\ \left.+2{\tilde{\omega }}^{\phi }\;\sin\left(\frac{\pi \phi }{2}\right)\cos\;\left(\tilde{\omega }\tau_{1}\right)-2{\tilde{\omega }}^{\phi }\;\cos\left(\frac{\pi \phi }{2}\right)\sin\;\left(\tilde{\omega }\tau_{1}\right)-\sin\;\left(\tilde{\omega }\tau_{1}\right)\right)\text{.} \end{array}$$
